# Exploration of the intelligent-auxiliary design of architectural space using artificial intelligence model

This article has been retracted.

**DOI:** 10.1371/journal.pone.0282158

**Published:** 2023-03-03

**Authors:** Hongyu Li, Qilong Wu, Bowen Xing, Wenjie Wang

**Affiliations:** School of Civil Engineering and Architecture, Shandong University of Science and Technology, Qingdao City, China; TU Wien: Technische Universitat Wien, AUSTRIA

## Abstract

In order to carry out a comprehensive design description of the specific architectural model of AI, the auxiliary model of AI and architectural spatial intelligence is deeply integrated, and flexible design is carried out according to the actual situation. AI assists in the generation of architectural intention and architectural form, mainly supporting academic and working theoretical models, promoting technological innovation, and thus improving the design efficiency of the architectural design industry. AI-aided architectural design enables every designer to achieve design freedom. At the same time, with the help of AI, architectural design can complete the corresponding work faster and more efficiently. With the help of AI technology, through the adjustment and optimization of keywords, AI automatically generates a batch of architectural space design schemes. Against this background, the auxiliary model of architectural space design is established through the literature research of the AI model, the architectural space intelligent auxiliary model, and the semantic network and the internal structure analysis of architectural space. Secondly, to ensure compliance with the three-dimensional characteristics of the architectural space from the data source, based on the analysis of the overall function and structure of space design, the intelligent design of the architectural space auxiliary by Deep Learning is carried out. Finally, it takes the 3D model selected in the UrbanScene3D data set as the research object, and the auxiliary performance of AI’s architectural space intelligent model is tested. The research results show that with the increasing number of network nodes, the model fitting degree on the test data set and training data set is decreasing. The fitting curve of the comprehensive model shows that the intelligent design scheme of architectural space based on AI is superior to the traditional architectural design scheme. As the number of nodes in the network connection layer increases, the intelligent score of space temperature and humidity will continue to rise. The model can achieve the optimal intelligent auxiliary effect of architectural space. The research has practical application value for promoting the intelligent and digital transformation of architectural space design.

## 1. Introduction

The success of modern architecture does not depend entirely on the creation of modern artistry but on the development of the material foundation. That is, more powerful industrial production technology is due to the improvement of material productivity brought about by the development of industrial technology [1–3]. Similarly, the rapid development of prefabricated buildings largely depends on technological progress in the entire assembly process. In other words, the progress of architectural design often depends on some innovative development outside of architecture. At present, the combination of Artificial Intelligence (AI) and the computer field is a huge leap. However, the intersection of neural networks and architecture design is not much, and they are basically focused on the engineering technology of architecture. This provides an opportunity for the combination of AI and architectural design. Thus, combining traditional architectural design with advanced AI will provide a new development opportunity.

In the era of AI, communication and discussion between architectural designers are essential sources to stimulate innovation, which is crucial to increase the necessary architectural intelligence space [4, 5]. Expanding the flexible space division according to the designer’s intention is necessary. There is a need to organize the space in an orderly form and maximize the Research and Development (R&D) space to adapt to the development of the AI industry. The common architectural intelligent space of the R&D office can meet the uncertain needs of industries and enterprises related to AI. Thus, it improves the operation efficiency of the park and promotes regional economic development. The current technical development background shows that the effective combination of AI and architectural space design can meet different individuals’ architectural space design needs [6].

In recent years, with the development of the AI industry and its extensive applications, AI technology has played a great role in architectural design and promoted the development of the architectural design. In the process of intelligent auxiliary design of architectural space, some scholars have expounded on the basic principles and conceptual methods of architectural design by the graphic method. They emphasize that space is an important means of architectural design, including how to organize the relationship between space and form. According to the introduction of meta-cosmic architecture, researchers proposed to pay attention to the promotion of the plot and the creation of large scenes. More attention has been paid to external modeling without considering the internal space. Compared with the traditional physical architectural space design and virtual game scene design, this design only provides a relatively simple and open indoor space. In the design process, the design time cycle is too long, and the design purpose of using the space ontology to interact with players at a higher level is not achieved so users feel less about the game space.

AI assists in the generation of architectural intention and architectural form, mainly supporting academic and working theoretical models, promoting technological innovation, and thus improving the design efficiency of the architectural design industry. AI-aided architectural design enables every designer to achieve design freedom. At the same time, with the help of AI, architectural design can complete the corresponding work faster and more efficiently. With the help of AI technology, through the adjustment and optimization of keywords, AI automatically generates a batch of architectural space design schemes. Designers can select the scheme from the options generated by AI learning with the most consistent design concept, area, and other actual parameters to deepen AI designs. In the process of architectural design, AI can assist designers to use different methods to create design and test models on-site, saving time and manpower. At the same time, AI can make work in the engineering field more efficient, save time for construction projects, improve work efficiency, and promote the development of the architectural design.

The optimization design of the architectural space is studied based on AI intelligent auxiliary model. The research aims to improve the intelligent level of architectural space design through AI auxiliary design. The main logical framework of this work is as follows. Section 1 introduces the development background of modern architectural design and AI models. Section 2 sorts out the recent literature on AI models and intelligent auxiliary design of architectural space. Then, Section 3 establishes the architectural space intelligent auxiliary system by analyzing the semantic network and architectural space structure. Section 4 analyzes the model’s performance by comparing the model’s building design error and accuracy loss. In Section 5, the research conclusion is drawn through systematic analysis and discussion. The research has practical reference value for promoting the deep integration of AI and architectural space model.

## 2. Literature review

### 2.1 Research progress of AI models

Based on the recent research on AI and Meta-Heuristic Optimizer (MHO), Jaafari et al. (2019) [7] evaluated the utility diagram of natural disaster intelligent hybrid integrated modeling based on a neuro-fuzzy system and MHO. The potential deviation inherent in the overfit single integrated model was overcome using four MHO to optimize the algorithm parameters. The results offered practical reference value for reliable estimation of the relative probability of natural disasters. Kuzior et al. (2019) [8] studied the possibility of sustainable development of organizations based on the combination model of AI. The research provided the theoretical and methodological background of organizational change and development and determined the possibility of applying AI technology in organizational functions. The results warranted the application of neural networks to intelligent organizational development management. Developing a combination model of AI for organizational development decision-making has been explored. Soni et al. (2019) [9] used AI models to predict the amount of urban solid waste. Comparing different models showed that accurate prediction of the amount of urban solid waste facilitated scholars to design and operate effective waste collection systems. Arrieta et al. (2020) [10] studied the concepts, classifications, opportunities, and challenges of responsible AI and proposed and discussed the latest classifications related to the interpretability of different machine learning models. Consequently, AI would promote the privacy and security of machine learning models. Lv et al. (2020) [11] studied the credibility of the industrial Internet of Things system based on artificial intelligence and studied building an evaluation framework based on machine learning knowledge. Online ranking algorithms were introduced as means of real-time analysis and evaluation of online data. The influencing factors of attack defense resources and the dynamic process of distributed cooperative control were obtained through simulation analysis. The outcome had practical reference value for promoting the development of the new generation network information physical system under the distributed cooperative control mode.

In addition to the application of artificial intelligence models in the industrial Internet of Things (IoT) systems, they are also widely used in medical testing and health care. For instance, Schneider et al. (2020) [12] reflected on drug design in the era of AI and introduced the significant challenges of different international expert groups on AI-produced small molecule drugs and the methods to solve these problems. As a result, AI methods presented new challenges not only for the scientists involved but also for the biopharmaceutical industry and its established processes for discovering and developing new drugs. Peng et al. (2021) [13] studied the AI model-assisted thyroid nodule diagnosis process based on the Deep Learning approach. They developed a deep AI model to distinguish malignant tumors from benign thyroid nodules. Apparently, integrating AI into thyroid nodule management effectively improved tumor identification accuracy. Lv et al. (2021) [14] examined AI based on industrial cyber-physical systems. Four modules based on detection, control, execution, and communication were chosen to study autonomous and flexible access to information. Testing and evaluating found that the effectiveness and robustness of the designed system were high. The research provided a theoretical basis and practical reference for developing the intelligent architectural industry. Elsheikh et al. (2022) [15] used a gradient-based optimizer to model the ultrasonic welding of polymers for AI models. Compared with other models, the proposed model had the highest determination coefficient and the lowest Root Mean Square Error (RMSE), Mean Relative Error (MRE), and variance coefficient. This indicated that the proposed scheme’s accuracy was higher than other test models. Kim et al. (2022) [16] employed AI models to assess Hepatocellular Carcinoma (HCC) risk in patients with chronic hepatitis B in Korea and the Caucasus. A risk-scoring model was developed to predict the risk of HCC in patients with chronic hepatitis B. As a result, the AI model provided the best risk prediction ability.

To sum up, the current research on the intelligent auxiliary model of architectural space has made many breakthroughs at many levels. Many strategies for the high-tech building industry and park design have been proposed. In general, no comprehensive design description has been made of the specific architectural model of AI. Therefore, the deep integration of AI and architectural space intelligent auxiliary models requires flexible design according to the actual situation.

### 2.2 Intelligent auxiliary design and research of architectural space

On the intelligent auxiliary model of architectural space, Zhao et al. (2018) [17] used AI and regression analysis to study the hybrid prediction model of office buildings’ dynamic cooling and heating load. Sensitivity and correlation analyses were used to select input variables and evaluate dynamic load prediction in different time ranges. The results showed that the proposed method realized high-precision dynamic load forecasting in different time ranges. Guo et al. (2018) [18] studied the user-centered semantic IoT technology for smart cities and used a new algorithm of AI semantic IoT hybrid service architecture to integrate heterogeneous IoT devices to support intelligent services. The results showed that the proposed architecture was supported by semantics and AI technology, flexibly connecting heterogeneous devices. Tushar et al. (2018) [19] innovated the IoT for green building management through low-cost sensor technology and AI. It was revealed that the IoT could collect and monitor large amounts of data from different aspects of the building and feed the data to the processor of the management system. At the same time, the system reduced the energy consumption of buildings by studying how human activities affect the energy use information of buildings. The finding could be used to design energy-saving measures. Guo et al. (2019) [20] reviewed the application of AI in smart homes and clarified the function and role of AI in smart homes through a literature review and product review. The research determined the application status of AI in smart home products and its usage in individual households. It was observed that smart homes would pay more attention to the interaction between people and the environment in the foreseeable future, making the building more sustainable and personalized. Yigitcanlar et al. (2020) [21] studied the contribution and risk of AI in the construction of smart cities and provided insights on how AI contributes to the development of smart cities. The systematic literature method was chosen. Literature results were divided into the main dimensions of smart city development. Their summarization had practical reference value for improving the service construction level of smart cities.

In addition to developing architectural space technology in smart cities, Ngarambe et al. (2020) [22] studied the application of AI methods in architectural thermal comfort prediction. Optimizing traditional building control methods showed that achieving a balance between reducing building energy use and providing sufficient comfort is a major challenge. Kua et al. (2021) [23] studied computer and IoT technology, from satellite-aided computing to digitally enhanced space life. It reviewed the latest development in the IoT and the aerospace industry. The results showed that the rapid development of IoT technology provided opportunities for space exploration. Merabet et al. (2021) [24] studied the intelligent building control system for thermal comfort and energy saving. A comprehensive understanding of the complexity of providing thermal comfort in buildings was achieved in an energy-efficient manner. The results showed that the application of AI technology and personalized comfort model saved energy by an average of 21.81% to 44.36%. It increased user comfort perception by an average of 21.67% to 85.77%.

To sum up, the problems of AI in architectural design have changed over time, and some problems have not been solved, but this cannot stop people’s enthusiasm for exploration. Since the 21st century, the Internet has become increasingly popular. The computing power of computers has become increasingly intense, and the amount of data people can store has increased. AI models can enable more system optimization operations for the intelligent auxiliary design of architectural space.

## 3. Research on architectural space intelligent assistant system based on AI deep learning model

### 3.1 Semantic network and analysis of the architectural spatial structure

In the deep learning model, multi-layer sensors can simulate heterogeneous logic in neural networks [25, 26] and have great potential for neural network applications in speech recognition, image processing, automobile driving, and other fields. Many multimedia experts believe that neural networks can lend well to extremely complex problems. In order to shape the architectural structure, the real structure inside the architectural space must be explored. Thereby, the different crossing paths generated by the architectural space can be illustrated; that is, the space path. There are certain constraints between the interior and exterior of architecture. The design of architectural space is actually the interpretation of the space path. Designing more public sidewalks is the goal of designers. Vertical area units are typically used to study space paths. When the research reaches a specific area, a unique spatial form is related to the formation of machines, and machines have different value orientations. Therefore, optimizing the design strategy of architectural space through machine learning and semantic network can improve the efficiency of architectural space design and reduce the cost. The intelligent auxiliary design structure of the semantic network and architectural space is sorted out. The overall structure design is shown in Fig 1.

**Fig 1:** Intelligent auxiliary design structure of architectural space.

### 3.2 Architecture and design of architectural space design model

The semantic model is the basis for effectively solving complex spatial problems and researching scientific and reasonable architectural space design methods. The semantic model of space design is a more intuitive analysis method, more convenient for solving problems. It is a more accurate internal factors analysis and further standardized space design [27]. New methods can be devised for architectural space design by combining semantic networks with architectural space design theory. They are easier to understand some architectural functions and use a unified space connected to a whole in a continuous order from the beginning to the end. This form of spatial combination is generated by using paths connected through space with clear directional relationships. When designing architectural space, the design method of functional area is developed according to different user requirements. The internal space is divided into adjacent space shapes of different sizes to meet customers’ different purposes effectively. In addition, the overall design process of architectural space is analyzed. The data transmission process of the architectural space model is shown in Fig 2:

**Fig 2:** Data transmission process of the architectural space model.

### 3.3 Analysis of the overall function of architectural space design

In the structural design of complex architectural space [28], function and shape correspond to the relationship between building unit areas to a certain extent. The transition from a single room to a whole space is reflected not only in the room’s functional requirements but also in the shape of the building. The expression of space design and function is usually used for buildings with high functional requirements. From the completion of the technical proposal to the construction technology implementation, each stage of the design is closely related to the space design strategy. Based on the above analysis, the overall structure of the architectural space design is analyzed, and the structure is shown in Fig 3:

**Fig 3:** Overall function and structure diagram of architectural space design.

### 3.4 Data processing and model analysis

This work focuses on the intelligent auxiliary design of architectural space by Deep Learning in AI. In order to ensure that Deep Learning conforms to the 3D characteristics of architectural space from the source of data, the 3D model from the UrbanScene3D data set is selected as the research object (UrbanScene3D contains 1.43TB of data in total, https://vcc.tech/UrbanScene3D. It provides classified download and related description of relevant data of UrbanScene3D and supports three download methods of Google Drive, Dropbox, and Baidu Cloud. Then, a data-driven way is needed to understand and process 3D data, namely 3D Deep Learning. 3D data are more difficult to apply to Deep Learning than 2D data. As an illustration, 2D graphics can be easily converted into matrix data, while 3D data becomes very difficult to process. Therefore, it is necessary to select the expression form of 3D data. In modeling, images from multiple angles represent objects with depth channels through which spatial data features are described. The specific experimental environment of the model is analyzed, and the environment configuration is shown in Table 1:

**Table 1:** Experimental environment settings.

Parameters	Specific information
Operating System (OS)	Windows10
Central Processing Unit (CPU)	i7-7700
CPU main frequency	3.60GHz
Random Access Memory (RAM)	16GB
Main chipset	Intel B250
CPU platform	Intel
Maximum memory	64GB
Graphics Processing Unit (GPU)	NVIDIA GeForce GTX 1080×4
Hard disk	50GB

In addition, as for the spatial intelligent auxiliary performance of the model, indicators such as architectural design error, building accuracy loss value, model fitting degree, prediction value conformity, space temperature score, and space humidity intelligence score are used for intelligent evaluation of the model. According to the ISO (International Organization for Standardization) 7730 standard, a PMV (Predicted Mean Vote) = 0.5 means the buildings’ function complies with comfortable feeling and energy-saving. The GB50019-2003 defines PMV = 1.0 as a building with comfortable health and energy-saving functions. The design error of the architectural model can be calculated by Eq (1):

$$Error=bias+V+B_{E}$$ (1)

In Eq (1), *bias* represents bias, which describes the fitting ability of the model. *V* denotes the variance, which is the impact of data disturbance. *B*_*E*_ is the error of the data itself. The architectural model’s design accuracy can be calculated by Eq (2):

$$P=\frac{TP}{TP+FP}$$ (2)

In Eq (2), *P* means Precision. *TP* indicates the True samples predicted as True by the model in the test samples. *FP* means the False samples predicted as True by the model in the test samples. The model fitting degree can be obtained by the cross-entropy algorithm of the Loss function. The space temperature is calculated by Eq (3):

$$t_{sa}=t_{e}+\frac{\rho I}{\alpha_{e}}$$ (3)

In Eq (3), *t*_*sa*_, *t*_*e*_, and *ρ* represent the comprehensive temperature, the outdoor air temperature, and the solar radiation absorption coefficient (set to 1.6), respectively. The outer surface heat transfer coefficient is set to $23.26\frac{W}{\left(m^{2}∙K\right)}$. Space humidity is calculated by Eq (4):

$$RH=\frac{P_{w}}{P_{ws}\left(T\;\;dry\right)}\times 100\%$$ (4)

In Eq (4), *RH* represents the spatial relative humidity. *P*_*w*_ and *P*_*ws*_(*T*) the absolute humidity and the saturated vapor pressure.

The model performance is analyzed and compared after sorting out the data. The structure of the proposed AI model is analyzed. The spatial intelligent auxiliary design process of the AI model is shown in Fig 4:

**Fig 4:** Spatial intelligent auxiliary design process of AI model.

## 4. Results and discussions

### 4.1 Data evaluation of architectural design error and accuracy loss of the model

In order to compare the auxiliary performance of AI-based architectural spatial intelligent models, the statistical data of building design errors of the test model and the training model are compared. Based on the method of point cloud visualization and under the framework of Deep Learning, the neural network is used to evaluate the auxiliary performance of the AI architectural space intelligent model. The trend of architectural design error of different architectural space auxiliary models with the increase of node number is shown in Fig 5.

**Fig 5:** The variation trend of architectural design error of different architectural space auxiliary models with the increase of node number.

According to Fig 5, when the network nodes increase, the actual design error of the test model and training model for architectural space intelligent auxiliary design will decrease significantly. When the number of connected nodes in the network is 20, the architectural design error of the training model is 0.49, and the architectural design error of the test model is 0.75. When the number of network nodes increases to 100, the architectural design error of the training model decreases to 0.25; the architectural design error of the test model is reduced to 0.40. Therefore, by adjusting the number of network nodes in the model, the design accuracy of the model is greatly improved, and the architectural design error can be reduced. The changing trend of accuracy loss of different architectural space auxiliary models with the increase of node number is shown in Fig 6.

**Fig 6:** The changing trend of accuracy loss of different architectural space auxiliary models with the increase of node number.

As per Fig 6, in different architectural space auxiliary models, the accuracy loss decreases with the increase in network nodes. When the number of network layer nodes is 20, the accuracy loss of the training model is 0.78, and the accuracy loss of the test model is 0.85. Besides, the accuracy loss will decrease significantly after the number of network layer nodes reaches 60. When the number of nodes is 60, the loss of accuracy of the architectural space auxiliary model on the training set is 0.7. When the number of nodes increases to 80, the accuracy loss on the training set space auxiliary model can be reduced to 0.55. When the number of nodes increases to 100, the accuracy loss on the training and test sets is the minimum. At this time, the accuracy loss of the training set model and the test set model is 0.25 and 0.4, respectively. Therefore, the accuracy performance of the model can be optimized by adjusting the number of network nodes.

### 4.2 Changing trend of model fit and predicted value fit

The model fitting degree of the architectural space model design and the conformity of the predicted value of the model is evaluated. The fitting degree trend of different architectural space auxiliary models with the increase in network nodes is shown in Fig 7.

**Fig 7:** The trend of the model fitting degree of different architectural space auxiliary models with the increase of the number of network nodes.

Apparently, in different architectural space auxiliary models, as the number of network nodes increases, the model fitting degree on the test data set and the training data set decreases. When the number of network nodes is 20, the model fitting degree on the test data set and the training data set is the largest: 0.7 and 0.35. When the number of network nodes increases to 100, the model fitting degree of the test data set decreases to 0.3, and the model fitting value of the training data set is reduced to about 0.2. Overall, the fitting curve of the comprehensive model shows that the intelligent design scheme of architectural space based on AI is superior to the traditional architectural design scheme. The trend of the compliance of the prediction values of different architectural space auxiliary models with the increase in the number of network nodes is shown in Fig 8.

**Fig 8:** The trend of the compliance of the prediction values of different architectural space auxiliary models with the increase of the number of network nodes.

Fig 8 suggests that under different architectural space design schemes, the conformity of the predicted value of the model will fluctuate. When the number of network nodes is 20, the conformity of the predicted value of the test model is 0.51, while the conformity of the predicted value of the training model is 0.18. In addition, when the number of network nodes increases to 100, the test model’s predicted value decreases to 0.16, while the training model’s predicted value is 0.12. Therefore, For the prediction value compliance performance of the model, it is necessary to adjust the number of network nodes within the range of 20~80 to ensure the optimal auxiliary design performance of the model.

### 4.3 Change trend of model space temperature score and space humidity intelligent score

The internal temperature and humidity scores are very important for architectural space design. The training model’s space temperature score and space humidity score data are collected and compared with the test model’s space temperature score and space humidity score data. The changing trend of the spatial temperature score and the spatial humidity intelligence score of the training model data in the spatial intelligent auxiliary model is shown in Fig 9.

**Fig 9:** Changing trend of spatial temperature score and spatial humidity intelligent score of training model data in the spatial intelligent auxiliary model.

Fig 9 shows that in the spatial intelligent auxiliary model design process, the temperature and humidity scores in the architectural space will fluctuate due to the change in the number of nodes. When the number of nodes is 20, the intelligent score of space temperature is 57.5, and the intelligent score of space humidity is 45. Then when the number of network nodes is 120, the intelligent score of space temperature increases to 67. The intelligent score of space humidity is 50. Therefore, with the increase in the number of nodes in the network connection layer, the intelligent score of space temperature and humidity will continue to rise, and the model can achieve the optimal intelligent auxiliary effect of architectural space. The changing trend of the spatial temperature score and the spatial humidity intelligent score of the test model data in the spatial intelligent auxiliary model is shown in Fig 10.

**Fig 10:** Changing trend of spatial temperature score and spatial humidity intelligent score of test model data in the spatial intelligent auxiliary model.

Evidently, compared with the training model, the space temperature score and space humidity score of the test model in the spatial intelligent auxiliary model are lower. When the number of network nodes is 20, the space temperature score of the model is 35, while the space humidity score of the model is only 12. When the number of network nodes increases, the test model’s space temperature and humidity scores will climb up. When the number of nodes is 80, the intelligent score of space humidity is the highest, and the model’s intelligent score of space humidity is 47. When the number of nodes is 100, the intelligent score of space temperature is the highest, and the model’s intelligent score of space temperature is 80. Therefore, selecting the appropriate number of network nodes for different space auxiliary models is necessary to optimize the model’s performance.

## 5. Conclusions

Today, countries worldwide are developing AI technology, but there is little research on the combination of architecture and AI. This work analyzes the course of architectural intelligent auxiliary design. It constructs the auxiliary model of architectural space design from the modular and computer-auxiliary design perspective. Based on the semantic network and the analysis of architectural space structure, the data transmission process of the architectural space model is analyzed through the architecture and design of the architectural space design model. Secondly, to ensure compliance with the three-dimensional characteristics of the architectural space from the data source, the intelligent design of the architectural space auxiliary by Deep Learning is carried out based on the analysis of the overall function and structure of space design. Finally, it takes the 3D model selected in the UrbanScene3D data set as the research object, and the auxiliary performance of the AI-assisted architectural space intelligent model is tested. The research results show that (1) under different architectural space design schemes, the consistency of the predicted values of the model will fluctuate. (2) The fitting degree of different architectural space auxiliary models between test data sets and training data sets is reduced. (3) In the process of intelligent auxiliary model design, the temperature and humidity scores in the architectural space will fluctuate with the number of nodes. Hence, by adjusting the number of intelligent network nodes in different architectural space auxiliary models, the design accuracy of the model has been greatly improved. The fitting curve of the comprehensive model shows that the intelligent design scheme of architectural space based on AI is superior to the traditional architectural design scheme. With the increase in the number of nodes in the network connection layer, the intelligent score of space temperature and humidity will continue to rise. The model can achieve the optimal intelligent auxiliary effect of the architectural space. Last but not least, there are some deficiencies in the research. The main deficiency is that the research on the internal functional zoning of architectural space is not perfect. In future research, it is necessary further to deepen the information structure database of the architectural semantic network and further optimize the intelligent auxiliary strategy of architectural space by using the Deep Learning model.
